This article has been retracted.

# Mutual Knowledge Analysis of Music Online Communication and Contemporary People's View of Music Based on Gray Correlation Analysis and Knowledge-Driven

**DOI:** 10.1155/2022/3942427

**Published:** 2022-08-04

**Authors:** Xiaojing Niu

**Affiliations:** College of Music and Dance, Huaihua University, Huaihua 418000, Hunan, China

## Abstract

With the operation and development of social economy, the emergence of network technology has caused a series of changes in contemporary music media and people's conception of music. A series of transformations have occurred. The article focuses on music network communication and the public's music concept and elaborates on the transformation of its concept and its influence, aiming to lay a good foundation for the development of music network communication through the study of the problem.

## 1. Introduction

With the development of social and cultural pluralism, music dissemination gradually shows the development of time, and modern music dissemination methods gradually change from CD and tape dissemination to forms of network dissemination [1]. This kind of dissemination method gradually expands people's choice of music so that people can more intuitively experience the potential artistic value of music while analyzing the emotional content of music [2].

Music communication is a unique and cutting-edge discipline in contemporary times. Music communication is formed on the basis of music communication research. This shows that people are beginning to understand music communication rationally while recognizing the phenomenon of music communication and spreading music culture. This phenomenon of music communication is not a narrow media phenomenon that we simply understand today. The phenomenon of musical communication is a broad, macro, and historical phenomenon.

The analysis of network transmission mode reveals that music data are mainly stored in digital format on the network, and users can restore music data through network equipment. Since the network is a whole, music data in the network environment can be disseminated in various service forms [3]. First of all, most network music dissemination in China is free; as long as users have network terminals, they can access music resources on the network, and listeners can also download and collect music and repeat and listen to it, which makes the scope of music dissemination more extensive and promotes the dissemination and development of music [4]. Secondly, network transmission has freedom, network environment has the form of resource sharing, and people can get music without the restriction of geography, time, and so on, thus providing a broader space for the spread of music [5]. Again, music producers can collect feedback from users on network platforms and adjust the production style of music through analysis of opinions, thus providing a good foundation for the development of music culture [6]. Finally, the information technology of the Internet fully demonstrates a wide range of music dissemination channels and diversity of information to a certain extent. Using the Internet as a basic innovation tool, it can realize the timely dissemination of music content and, at the same time, make people's information access concept change [7]. At the same time, in the network environment, the dissemination of information is virtual and massive, in which digital information technology and music content provide an effective basis for the generation and reproduction of information [8]. The development of network technology has brought great convenience to people's life and entertainment. Spreading music through the network can also provide listeners with the freedom to choose music and get people's recognition and acceptance. People who listen to music can also become producers. This new way of music transmission has many advantages, but everything has two sides, so it also has limitations. We should create a good network environment and innovate traditional music, promoting the development of music culture.

## 2. Related Work

Music communication is a cross-cutting field between musicology and communication science. In [9], music communication is studied from a disciplinary point of view, and the object of study, research paradigm, and basic theoretical models are defined, and popular music symbols, modes of communication, and media are systematically discussed. In addition to the five elements required for music communication based on the 5 Ws theory of communication [10], Cegarra-Navarro et al. also review the history of the development of communication in China and conclude that future development of communication should tend to deepen content and diversify branches, taking the emergence and development of music communication as an example [11]. Using a sociological perspective, Trunfio and Campana introduce concepts of production, audience, and dissemination in communication and grasp macroscopic and fluid music phenomenon as a whole, taking into account real-life phenomena and examples [12]. In his book “A Course in Sociology of Music,” von Rueden et al. devoted a chapter to music communication on the Internet and proposed six characteristics of music communication on the Internet [13]. In his work “Theory of Spiritual Communication,” Mazzucchelli et al. discuss literature as a form of communication and includes music communication in the category of literary communication [14]. In their study of music from the perspective of communication, they analyzed similarities and differences between music and music communication, and sorted out the evolution from the sociology of music to the study of music communication. In this paper, we explain music transmission in terms of the temporal nature of music symbolic transmission, arguing that the length and spatial structure of sound reflect the length of music transmission, which can only be measured in one direction. In other words, the process of music transmission is a linear process, and music embodies the quality of time in the process of transmission [15].

However, in the process of Internet operation, music dissemination in the network environment has led to a certain change in the public's perception of music, and there are corresponding opportunities and challenges in this transformation process [16]. For online communication, the music form is different from traditional music. Therefore, in this paper, while exploring music network communication, we systematically analyze the public's music concept, aiming to realize comprehensive improvement of the public's music concept and the inheritance and development of music culture [17].

## 3. Architecture

The development of the economy is an important material premise for the change in music dissemination in the Internet era. More and more high-tech products such as computers, MP3s, and music cell phones are consumed by the general public. Only with these carriers can changes in music dissemination in the Internet era be realized [18–20]. Similarly, only with the continuous development of the economy, human beings will pursue higher-level spiritual needs after their basic material life is guaranteed (as shown in Figure 1). Only after lower-level needs are satisfied, higher-level needs will be required.

He believes that there are two main types of music transmission, one of which is the “live” mode of music transmission, in which transmitter and recipient interact and share music in the same space and time, with the stage as the center of the transmission process. The dissemination model is shown in Figure 2.

The other is the “mediated” mode of transmission, in which the transmitter and the recipient interact and share music across time and space, with the medium as the center of the transmission process, and even copy and feedback. The transmission model is shown in Figure 3.

In 1990, Devereux and Bauer-Lokić proposed the ripple effect theory from the perspective of the relationship between mass communication media, audience, and society. In their book “Theories of Mass Communication,” they proposed that communication effects are mainly expressed in three structural forms: cognitive effects, emotional effects, and behavioral effects. From a macroscopic perspective, there are five levels: personal, interpersonal, organizational, systemic, and social. The effect of the media is like ripples produced by a stone thrown into a pond, spreading from center to surroundings in a specific process: personal communication effect layer, interpersonal communication effect layer, organizational communication effect layer, system communication effect layer, and social communication effect layer. If the process of media communication is described as a huge system, then any change in the effect of any level of communication will affect the change of the whole system, as shown in Figure 4.

Mp3, cell phones, iPads, computers, and other mobile devices have liberated listening range of public, allowing more songs to gain opportunity to “make a name for themselves,” but this does not mean that living conditions of musicians have become better because Chinese people have not yet developed habit of paying for listening, and income of musicians does not increase with rise of hits, as shown in Figure 5.

Microblogs are multilayered, and information is spread many times through “nested followers,” expanding the spread of information and forming a fissile spread. In practice, information about an independent musical work may be processed and disseminated by several Weibo users at the same time from similar or different perspectives, forming a larger dissemination network. Take video content of independent musician Xie Chunhua's adaptation and cover of Chen Hongyu's original work “Ideal Sanshun” as an example; there are nearly 90 Weibo original blog posts with similar content using the same video editor, as shown in Figure 6.

Xinzhou Xie of Peking University pointed out that the process of network communication is very complex and it is difficult to elaborate on the whole process, so he drew on German scholar Maletzke's systematic model of mass communication process to build a specific model from the perspective of a communicator to a node. He says that, in network communication, a process does not only reach a node and generate feedback but also reach other nodes through a node to achieve wider dissemination. He calls this model a “propagation model with respect to one node” (see Figure 7).

Drawing on the “propagation model relative to a node” model, this paper attempts to construct a microblog-based independent music propagation model (see Figure 8), eventually forming a wide information dissemination network.

As shown in Figure 9, solid line indicates the direction of information dissemination in WeChat, and a dashed line indicates the direction of information feedback. User A and user B are ordinary users of WeChat, and user A, who is a “friend” of WeChat, filters and processes independent music-related information from various channels and then delivers information to user B's WeChat through the WeChat client. User B chooses to receive information from User A or ignore it on his WeChat client. Because of the one-to-one interpersonal communication characteristics of WeChat and “strong relationship” network between two parties, User B usually reads messages rather than ignores it. In the initial stage of information transmission, user A is the transmitter and user B is the receiver; in the process of information feedback, the roles of the two parties are reversed. In the process of communication chat, transmission and feedback of information usually go through several cycles, until user A or B stops sending or receiving information; then, information temporarily stops spreading. Although there is less noise interference in one-to-one interpersonal communication, it is inevitable.

The macro information dissemination network of WeChat's circle of friends is constructed in the analysis of communication patterns of WeChat (see Figure 10).

The service number provides a business service and user management platform for enterprises and organizations; the enterprise number provides a mobile portal for enterprises or organizations, helping enterprises to establish connections with employees. Subscription numbers are a platform for independent musicians and their organizations or other individuals who operate related content to disseminate independent musical works and information, and they are a platform for accurate information dissemination and for independent musicians or labels to maintain relationships with users. Therefore, this section focuses on the distribution model of subscription numbers.  Figure 11 shows the independent music dissemination model of WeChat subscription number based on one node.

The diffusion of NetEase Cloud Music is based on a variety of channels, and users can find independent music that meets their needs through both active search and passive reception.  Figure 12 shows the diffusion network of music on the NetEase Cloud Music platform.

Figure 13 is a compilation of different ways in which users may manipulate independent music singles in the process of dissemination and the results of various manipulations.

## 4. Gray Correlation Analysis

It is a comparative analysis of similarity between series and reference series. This comparative analysis can be mathematically characterized as an analysis of similarity or proximity of curve shape or spatial distance. The more similar the curve shape or closer spatial distance is, the greater gray correlation is and the greater degree of correlation between the sequence and the reference sequence is. At present, gray correlation analysis has been widely used in various fields. However, many things described in matrix form (such as grayscale images and MFCC parameters of speech signals) can be compared by converting them into sequence form. However, a matrix is not a simple sum of several sequences, but a matrix has many characteristics that sequences do not have, such as eigenvectors and determinants. For such a problem, this paper proposes the concept of matrix gray correlation analysis in order to provide a new technical tool as a reference for the representation of things in matrix form.

**Proposition 1 .**

Set values of two-dimensional systems (such as two-dimensional airspace) to form mxn behavior matrix of the system:

(1) $$\begin{array}{c} X_{i}=\left[\begin{array}{cccc} x_{i}\left(1,1\right) & x_{i}\left(1,2\right) & \cdots & x_{i}\left(1,n\right)\\ x_{i}\left(2,1\right) & x_{i}\left(2,2\right) & \cdots & x_{i}\left(2,n\right)\\ \cdots & \cdots & \cdots & \cdots \\ x_{i}\left(m,1\right) & x_{i}\left(m,2\right) & \cdots & x_{i}\left(m,n\right) \end{array}\right]. \end{array}$$

Record *k*th line of the system behavior matrix, (*x*_*i*_(*k*, 1) − *x*_*i*_(*k*, 1), *x*_*i*_(*k*, 2) − *x*_*i*_(*k*, 1),…, *x*_*i*_(*k*, *n*) − *x*_*i*_(*k*, 1)), *x*_*i*_(*k*, 1), order:

(2) $$\begin{array}{c} s_{i}\left(k,\right)=\int_{1}^{n}\left(X_{i}\left(k,\right)-x_{i}\left(k,1\right)\right)\text{d}t,\;k=1,2,\ldots ,m. \end{array}$$

Record broken line in *L* line of the system behavior matrix:

(3) $$\begin{array}{c} \left(x_{i}\left(1,l\right)-x_{i}\left(1,l\right),x_{i}\left(2,l\right)-x_{i}\left(1,l\right),\ldots ,x_{i}\left(m,l\right)-x_{i}\left(1,l\right)\right), \end{array}$$

*x*_*i*_(*k*, 1), order

(4) $$\begin{array}{c} s_{i}\left(,l\right)=\int_{l}^{m}\left(X_{i}\left(,l\right)-x_{i}\left(1,l\right)\right)\text{d}t,\;I=1,2,\ldots ,n, \end{array}$$

where *x*_*i*_(*q*, *l*)*d*_*l*_=*x*_*i*_(*q*, *l*) − *x*_*i*_(1, *l*), *q*=1,2,…, *m*,  *l*=1,2,…, *n*. *D*_*n*1_ is column start point annihilation operator; *X*_*i*_*D*_*n*1_ is the column start point annihilation image of *X*_*i*_, recorded as

(5) $$\begin{array}{c} X_{i}D_{n1}=X_{i}^{n}=\left[\begin{array}{cccc} x_{i}^{,1}\left(1,1\right) & x_{i}^{,2}\left(1,2\right) & \cdots & x_{i}^{,n}\left(1,n\right)\\ x_{i}^{,1}\left(2,1\right) & x_{i}^{,2}\left(2,2\right) & \cdots & x_{i}^{,n}\left(2,n\right)\\ \cdots & \cdots & \cdots & \cdots \\ x_{i}^{,1}\left(m,1\right) & x_{i}^{,2}\left(m,2\right) & \cdots & x_{i}^{\prime n}\left(m,n\right) \end{array}\right], \end{array}$$

where *x*_*i*_^*l*^(*q*, *l*)=*x*_*i*_(*q*, *l*) − *x*_*i*_(1, *l*),  *q*=1,2,…, *m*.

**Definition 1 .**

Set system behavior matrix:

(6) $$\begin{array}{c} X_{i}=\left[\begin{array}{cccc} x_{i}\left(1,1\right) & x_{i}\left(1,2\right) & \cdots & x_{i}\left(1,n\right)\\ x_{i}\left(2,1\right) & x_{i}\left(2,2\right) & \cdots & x_{i}\left(2,n\right)\\ \cdots & \cdots & \cdots & \cdots \\ x_{i}\left(m,1\right) & x_{i}\left(m,2\right) & \cdots & x_{i}\left(m,n\right) \end{array}\right], \end{array}$$

*D*_1_ is a matrix operator, and

(7) $$\begin{array}{c} X_{i}D_{1}=\left(x_{i}\left(k,1\right)d_{1},x_{i}\left(k,2\right)d_{1},\ldots ,x_{i}\left(k,n\right)d_{1}\right)\;k=1,2,\ldots ,m, \end{array}$$

where *x*_*i*_(*k*, *p*)*d*_1_=*x*_*i*_(*k*, *p*) − *x*_*i*_(1,1),  *p*=1,2,…, *n*. Then, *D*_1_ is the uniform starting point annihilation operator and *X*_*i*_*D*_*n*1_ is the uniform starting point annihilation image of*X*_*i*_ and is recorded as

(8) $$\begin{array}{c} X_{i}D_{1}=X_{i}^{0}=\left[\begin{array}{cccc} x_{i}^{0}\left(1,1\right) & x_{i}^{0}\left(1,2\right) & \cdots & x_{i}^{0}\left(1,n\right)\\ x_{i}^{0}\left(2,1\right) & x_{i}^{0}\left(2,2\right) & \cdots & x_{i}^{0}\left(2,n\right)\\ \ldots & \ldots & \cdots & \cdots \\ x_{i}^{0}\left(m,1\right) & x_{i}^{0}\left(m,2\right) & \cdots & x_{i}^{0}\left(m,n\right) \end{array}\right], \end{array}$$

where *x*_*i*_^0^(*q*, *p*)=*x*_*l*_(*q*, *p*) − *x*_*j*_(1,1),  *q*=1,2,…, *m* and *p*=1,2,…, *n*.

**Definition 2 .**

et $X_{i}=\left[\begin{array}{cccc} x_{i}\left(1,1\right) & x_{i}\left(1,2\right) & \cdots & x_{i}\left(1,n\right)\\ x_{i}\left(2,1\right) & x_{i}\left(2,2\right) & \cdots & x_{i}\left(2,n\right)\\ \cdots & \cdots & \cdots & \cdots \\ x_{i}\left(m,1\right) & x_{i}\left(m,2\right) & \cdots & x_{i}\left(m,n\right) \end{array}\right]$ be behavior matrix of factor *X*_*i*_.

(9) $$\begin{array}{c} X_{i}D_{m22}=\left(x_{i}\left(k,1\right)d_{k},x_{i}\left(k,2\right)d_{k},\ldots ,x_{i}\left(k,n\right)d_{k}\right)=\left[\begin{array}{cccc} x_{i}\left(1,1\right)d_{m2} & x_{i}\left(1,2\right)d_{m22} & \cdots & x_{i}\left(1,n\right)d_{m2}\\ x_{i}\left(2,1\right)d_{m2} & x_{i}\left(2,2\right)d_{m22} & \cdots & x_{i}\left(2,n\right)d_{m22}\\ \ldots & \cdots & \cdots & \cdots \\ x_{i}\left(m,1\right)d_{m2} & x_{i}\left(m,2\right)d_{m2} & \cdots & x_{i}\left(m,n\right)d_{m22} \end{array}\right],\;k=1,2,\ldots ,m, \end{array}$$

where

(10) $$\begin{array}{c} x_{i}\left(k,p\right)d_{m2}=\frac{x_{i}\left(k,p\right)}{x_{i}\left(k,1\right)},\;x_{i}\left(k,1\right)\neq 0,\;p=1,2,\ldots ,n, \end{array}$$

where *d*_*m*2_ is row initialization operator, and *X*_*i*_*D*_*m*2_ is image of *X*_*i*_ under row initialization operator *D*_*m*2_, which is referred to as row initialization image for short.

**Definition 3 .**

Let $X_{i}=\left[\begin{array}{cccc} x_{i}\left(1,1\right) & x_{i}\left(1,2\right) & \cdots & x_{i}\left(1,n\right)\\ x_{i}\left(2,1\right) & x_{i}\left(2,2\right) & \cdots & x_{i}\left(2,n\right)\\ \cdots & \ldots & \cdots & \cdots \\ x_{i}\left(m,1\right) & x_{i}\left(m,2\right) & \cdots & x_{i}\left(m,n\right) \end{array}\right]$ be behavior matrix of factor *X*_*i*_, *D*_*n*2_ be matrix operator, and

(11) $$\begin{array}{c} X_{i}D_{n2}=\left(x_{i}\left(1,l\right)d_{k},x_{i}\left(2,l\right)d_{k},\ldots ,x_{i}\left(m,l\right)d_{k}\right)\\ =\left[\begin{array}{cccc} x_{i}\left(1,1\right)d_{n2} & x_{i}\left(1,2\right)d_{n2} & \cdots & x_{i}\left(1,n\right)d_{n2}\\ x_{i}\left(2,1\right)d_{n2} & x_{i}\left(2,2\right)d_{n2} & \cdots & x_{i}\left(2,n\right)d_{n2}\\ \cdots & \cdots & \cdots & \cdots \\ x_{i}\left(m,1\right)d_{n2} & x_{i}\left(m,2\right)d_{n2} & \cdots & x_{i}\left(m,n\right)d_{n2} \end{array}\right],l=1,2,\cdots ,n, \end{array}$$

where

(12) $$\begin{array}{c} x_{i}\left(q,l\right)d_{n2}=\frac{x_{i}\left(q,l\right)}{x_{i}\left(q,l\right)},\;x_{i}\left(q,l\right)\neq 0,\;q=1,2,\ldots , \end{array}$$

where *d*_*n*2_ is a column initializing operator, and *X*_*i*_*D*_*n*2_ is an image of *x*_*i*_ under column initializing operator *D*_*n*2_, which is referred to as the column initializing image for short.

## 5. Results

The development of the Internet and computers in China can be statistically investigated in many ways. One of them is the China Internet Information Center, which has been keeping an eye on its development. Detailed and continuous statistical surveys have been done on various aspects such as number of people accessing the Internet, their way of accessing the Internet, the number of computers accessing the Internet, the number of websites, and the age and education statistics of people accessing the Internet. The following is the statistical chart of users and computers in China from 2010 to 2021, as shown in Figure 14.

From Figure 14, we can see that Internet computers on the Internet have been increasing dramatically in the past 10 years. Especially since 2010, the number of Internet users has been increasing linearly, and the number of computers on the Internet has been growing rapidly since 2011. This shows that, in this short decade, especially after 2021, the Internet audience in China is growing rapidly and computers have become the main means for people to access the Internet. Conversely, it is the popularity of computers that makes the Internet an increasingly one of contemporary mass communication media.

As a new product of the information technology revolution, the rapid development of the Internet is growing exponentially. As of December 31, 2010, Chinese Internet users accounted for 23.2% of the world, 55.4% of Asia, 450 million broadband, 98.3% of fixed network penetration, and 3413 CN domain names nationwide. There are 3413127 CN domain names. According to the survey, China's personal Internet application index reached 57.6. Although the Internet Entertainment index is slightly lower than that in previous years, the utilization rate of online music, online games, and online video is still at a high level. Obviously, the Internet is becoming more and more important as a new medium for music communication activities (see Table 1).

In this paper, as an Internet user, we have done a general statistics and arrangement of online music resources on Internet. It is found that music culture in online media is mainly dominated by contemporary pop music culture, while Chinese folk music does not occupy a large share in comparison. The following is data from an online survey done by Kugoo, Xunlei, Baidu MP3, and Baidu posting bar to compare the status of resources of ethnic music varieties or by certain ethnic instruments, traditional repertoire, and performers, with the status of resources of pop music performers and repertoire: it should be noted that numbers in Tables 2–5 represent the number of music resources in terms of songs.

Figure 14 shows that pop music is prevalent on the Internet while traditional folk music resources are scarce. This paper argues that there are several reasons for this situation. First, the online audience has very limited resources of digitized folk music that can be disseminated on the Internet. Second, there is a serious imbalance of folk music in the overall environment of contemporary online music dissemination, and popular music has become the main force of music dissemination. Once again, in the era of mass communication, the spirit of entertainment has influenced media organizations and the general audience. Again, music professionals are not making full use of online media to take the initiative to fill the gap in online resources related to folk music and serious music. This is why it is important to try to establish a digital music sharing program with professional institutions as a unit, which is an effective solution to this problem.

## 6. Conclusions

In summary, the development of network technology has brought great convenience to people's life and entertainment, and the dissemination of music through networks can also provide listeners with the freedom to choose music. The article focuses on music network communication and the public's music concept as the focus of research and elaborates on the transformation of its concept and its influence, aiming to lay a good foundation for the development of music network communication through the study of problems, which is recognized and accepted by people, and people who listen to music can also become producers; this new way of music dissemination has many advantages, but there are two sides to everything, so it also has limitations, and it is necessary to create a good network environment, to innovate traditional music, and to promote the development of music culture.

## Figures and Tables

**Figure 1:** Hierarchy of needs theory.

**Figure 2:** Live music transmission mode.

**Figure 3:** Music “media” communication mode.

**Figure 4:** Ripple effect.

**Figure 5:** Analysis of development of online performance market.

**Figure 6:** Microblog independent music node propagation network.

**Figure 7:** Propagation mode of a node.

**Figure 8:** Independent music propagation mode of microblog relative to one node.

**Figure 9:** Wechat communication mode in context of instant messaging.

**Figure 10:** Macro information dissemination network of WeChat circle of friends.

**Figure 11:** WeChat subscription number propagation mode.

**Figure 12:** NetEase Cloud Music macro communication network.

**Figure 13:** NetEase Cloud Music micro propagation mode.

**Figure 14:** Development trend of computer network in China.

**Table 1:** Calculation of personal Internet application index in 2010.

Primary index	Secondary index	Tertiary indicators	Utilization rate (%)
Personal internet application index	Information access index	Network news	77.3
		Search engines	82.1
	Internet entertainment index	Network music	79.3
		Network game	66.6
		Network video	62.5
	Interactive participation index	Instant messaging	77.4
		E-mail	54.5
		Update blog	40.0
		Post and reply online	31.6
	Online consumption index	Online shopping	35.5
		Online payment	30.0
		Travel reservation	8.0

**Table 2:** Data list of traditional music varieties on different network platforms.

	Folk song	Traditional opera	National instrumental music	Quyi
KUGOO	230	7	18	6
Thunder	3862	201	80	8
Baidu mp3	105	413	5	168
Baidu tieba	578	638	2	158

**Table 3:** List of search data of representative musical instruments, representative tracks, and important performers.

	Erhu fiddle	Guqin	Pipa	Mei Lanfang	Beijing opera	Ji Shi Diao Youlan
Kugoo	120	8	20	3	44	4
Thunder	300	170	17	17	270	18
Baidu mp3	1360	435	67	173	2250	35
Baidu tieba	1080	589	665	620	4670	15

**Table 4:** List of pop music representative singers and representative songs search data.

	Jay Chou	Faye Wong	She	Mice love rice
Kugoo	355	353	420	115
Thunder	18620	15652	4800	1147
Baidu mp3	41000	11310	8750	4650
Baidu tieba	359460	32545	25357	8958

**Table 5:** Overview of data of various music resources on various network platforms.

	Kugoo	Thunder	Baidu mp3	Baidu post bar	Total
Folk song	230	3862	105	575	4772
Traditional opera	8	215	410	635	1266
National instrumental music	15	72	2	3	92
Traditional opera	6	6	168	152	333
Erhu fiddle	120	300	1360	1088	2868
Guqin	7	170	438	582	1197
Pipa	20	19	66	665	770
Mei Lanfang	4	14	170	620	810
Beijing opera	45	270	2250	1690	7255
Orchid in seclusion	3	18	34	13	67
Jay Chou	340	18640	41000	359460	419440
Faye Wong	355	15665	11300	32540	59860
She	422	4806	8760	353430	267418
Mice love rice	115	1155	5660	8965	15895

## Data Availability

The experimental data used to support the findings of this study are available from the author upon request.
